RETRACTED

# Energy-Efficient and Secure Opportunistic Routing Protocol for WSN: Performance Analysis with Nature-Inspired Algorithms and Its Application in Biomedical Applications

**DOI:** 10.1155/2022/1976694

**Published:** 2022-03-25

**Authors:** Deep Kumar Bangotra, Yashwant Singh, Nagesh Kumar, Pradeep Kumar Singh, Adegoke Ojeniyi

**Affiliations:** ^1^Department of Higher Education, J&K Govt., India; ^2^Department of Computer Science and Information Technology, Central University of Jammu, J&K, India; ^3^Chitkara University School of Engineering and Technology, Chitkara University, Himachal Pradesh, India; ^4^Department of Computer Science, KIET Group of Institutions, Delhi-NCR, Ghaziabad, India; ^5^Department of Computer Science, The Maldives National University, Maldives

## Abstract

Wireless sensor network (WSN) is made up of tiny sensor nodes. The application of WSN in diverse fields has seen a tremendous escalation in recent years. WSN applications are constrained by the limited set of computing resources possessed by the sensor nodes and the security aspects of data communication in the WSN. Many algorithms based on nature-inspired optimization (NIO) have been proposed in the past to optimize the issue of energy efficiency and security in WSN. In the proposed work, two opportunistic routing algorithms, i.e., intelligent opportunistic routing protocol (IOP) and trust-based secure intelligent opportunistic routing protocol (TBSIOP), are compared against two NIO algorithms developed for achieving energy efficiency and security in WSN for performance analysis. The performance is evaluated by simulating the algorithms on MATLAB and comparing the obtained results with existing ACO-based and PSO-based routing algorithms. It is observed that the TBSIOP outperforms the NIO-based algorithms in terms of energy efficiency, network lifetime, packet delivery ratio, end-to-end delay, and average risk level. All the parameters under consideration are recorded in the presence of a maximum of 50% malicious nodes for 25, 50, and 100 nodes' test cases. The increasing size of the network has a significant effect on the performance of TBSIOP, as the packet delivery ratio is close to 100%. Also, TBSIOP can easily avoid malicious nodes during the routing process as reflected from the results. This will improve the network lifetime of TBSIOP compared to other protocols. As far as the application of the work is concerned, it would be beneficial for smart healthcare services. It can also help in better communication during the sharing of data by providing energy-efficient services and keeping the network alive for a longer period.

## 1. Introduction

With the proliferation of microelectromechanical systems (MEMS) in the last decade, the mobile ad hoc network (MANET) has gained tremendous importance. These networks over a while have found their applications in almost every aspect of life. Wireless sensor networks (WSN) being a special type of network under ad hoc networks are composed of nodes that are not fixed for one location. WSN is made up of microsized sensor nodes which are capable of self-configuration. The WSN nodes are deployed randomly for observing and recording the physical phenomenon in locations that are mostly unreachable by humans. The function of these sensor nodes is dependent on constrained computing resources such as battery, storage, and processing capabilities [1]. A typical sensor node is capable of performing three basic operations in the sensor network. They have the ability to sense, transmit, and process the acquired data in the area of node deployment. In some scenarios, the sensor nodes are equipped with additional infrastructure for location detection and ensuring mobility in the network. Sensors are set in such a way that their capabilities, such as storage space, energy, and communication, are used effectively. Any sensor has a finite level of energy at first, but as the communication between nodes progresses, this energy is exhausted. Since the region under observation is normally unattended, the option to repair or restore sensor nodes does not exist. If a single node fails to perform its duty, the network can become unusable, and there will be a topology change. This scenario will lead to the reconstruction of network topology, and retransmission will take place in the network. As a result, in a WSN, there will be a reduction in the battery life of the sensor nodes, and consequently, the lifetime of the sensor network will be reduced. Therefore, energy efficiency and network longevity are the two prominent challenges present in the WSN that are to be addressed.

RETRACTED

Routing in WSN is a hot topic of study, with researchers looking for ways to improve WSN. Until now, energy-effective routing has been a significant hurdle to overcome. A protocol for data communication is necessary among nodes (routers) of a WSN to determine a path for data transfer in the network. Many energy-effective data communication protocols are configured to spread the energy load through all nodes, lowering power utilization in a WSN. Similarly, the security of the data transmitted over the sensor network is a significant challenge. Owing to the unrestricted wireless networking aspect of WSN and the restricted capabilities of nodes, maintaining security and confidentiality is a significant challenge [2]. Encryption and cryptographic keys are the most popular authentication mechanisms utilized in wireless networks. While encryption ensures anonymity, honesty, and authenticity, it comes at a high price in terms of energy and processing costs. Intrusion prevention technologies and trust-based protocols are better at detecting misbehaving nodes. The trust management paradigm is more flexible, scalable, and reliable than traditional protection mechanisms. By creating a trust relationship among sensor nodes, sharing and security services can be provided. Based on the computation of a node's confidence values, the trust model increases protection in an open network environment. Therefore, there are trust and reputation-based methods that offer lightweight solutions to address the challenge of security in WSN.

The real-world problems are divided into two types, i.e., deterministic and nondeterministic problems. Routing is one of the most difficult problems in WSN for which there is no deterministic solution. As a result, nature-inspired optimization (NIO) algorithms are used to present low-cost routes across a variety of options. Various routing algorithms have been created using swarm intelligence- (SI-) [2] related algorithms. SI can be seen as a link between programming approaches and swarm actions influenced by nature. The intelligent algorithms built on swarms can provide the best answers to real-world problems. The illustration for some of the most common SI-based optimization techniques available in the literature for routing is shown in Figure 1.

This paper describes some of the most popular nature-inspired optimization algorithms for addressing the challenge of routing and security in WSN to achieve energy-efficient and secure sensor networks. A comparative analysis of two protocols, i.e., IOP [3] and TBSIOP [4], with some of the NIO algorithms used for routing in WSN is presented in the subsequent sections. The primary goal here is to investigate present technological cutting-edge nature-inspired optimization strategies for data routing through WSN and to find effective routing approaches in a WSN. The main contribution of the paper is the comparative analysis of nature-inspired routing approaches and our previously proposed models IOP and TBSIOP. The significance of the proposed study in this paper can be considered as finding out the possibilities to use nature-inspired algorithms in WSN.

The rest of the paper is structured as follows. In Section 2, a detailed review of literature in respect of NIO swarm intelligence-based algorithms is presented. In Section 3, the important issues related to the routing are discussed, and Section 4 deals with the algorithms for the creation of forwarder node list, intelligent opportunistic routing protocol (IOP), and trust-based secure intelligent opportunistic routing protocol (TBSIOP). In Section 5, swarm intelligence- (SI-) based optimization techniques for routing in WSN are presented.  Section 6 discusses the experimental setup by simulating the protocols for comparative analysis in MATLAB, and Section 7 delivers the concluding remarks with the future scope of the research work.

RETRACTED

## 2. Literature Review

With the ever-evolving magnitude of WSN-based applications, the challenges in providing real-time optimal solutions are also increasing. The biggest issue with WSN which is discovered after a detailed study of literature is the ideal consumption of computational means available with the wireless sensor nodes. As these sensor nodes are always resource-constrained, the best utilization of their resources is of paramount significance for the survival and longevity of the sensor network. The sensor nodes are proficient in acquiring and transmitting the data with their respective modules. Moreover, it is the routing protocol that is to be applied for the transmission of data between sensor nodes and between the source node and the destination node, i.e., base station (BS). The challenge with routing in WSN is that it consumes a maximum of the node's resources during the communication process. Due to this significant amount of resource consumption during the transmission of data in the network, the longevity of the sensor node is affected and the overall functionality of the network is compromised. To address this challenge, NIO algorithms are presented in the literature. Their use in the literature has shown significant improvements in respect of energy utilization and network lifetime in the case of WSN. As a consequence, nature-inspired path optimization strategies play a critical role in a WSN, as efficient routing reduces energy usage and thereby increases network lifespan [5]. In a WSN, route optimization algorithms take into account not only path distance but also energy efficiency and network lifespan. Traditional routing methods are effective at achieving optimum solutions, but they use a lot of computing resources. Swarm intelligent algorithms and genetic algorithms have previously been seen to be effective for achieving efficient routing in a WSN. A considerable amount of analysis has been done in the past in sensor networks. The major focus of the research work in the past was related to traditional routing techniques in WSN [6–10]. Moreover, this section presents the latest research work in nature-inspired optimization algorithms for effective routing in WSN.

RETRACTED

The authors [12] have presented an exhaustive review about those routing protocols which employ swarm-based intelligence methods for addressing different issues in WSN. Though WSN has to deal with numerous issues like battery life, scalability, and complexity, these issues are to be considered while designing routing protocols for WSN. It has been ascertained by the researchers that out of numerous research issues in WSN, the application of swarm intelligence-based routing protocol controls at least one of the mentioned issues. Similarly, in another research paper, the authors described the use of swarm intelligence- (SI-) based data communication or routing protocols in WSN. A major chunk of research in SI draws its inspiration from the field of reverse engineering. The authors of this research paper conclude that these algorithms are adaptive, scalable, and robust and they are very similar to their corresponding natural systems, i.e., ant colonies and bee colonies. An exhaustive and important comparison between traditional and swarm intelligence-based routing protocols is presented in [13]. To understand the impact and have a yardstick for prospect work, different routing protocols provided in the analysis work are simulated again using a MATLAB-based simulator. It is also discovered from the study of literature that in [14], the authors have presented nature-inspired routing protocols specially designed for ad hoc and WSN. In the event of no-loop, energy-aware any-path routing, the authors conclude that ant colony optimization (ACO) and particle swarm optimization (PSO) have more encouraging performance. Path congestion, route optimality, and energy utilization are some of the metrics used to test the efficiency of these protocols. Different routing protocols in WSN which are developed using nature-inspired optimization techniques are presented in [15]. In this paper, network life is considered the most critical performance metric to measure the success of a network. This paper also describes the use of intelligent routing algorithms such as reinforcement learning (RL), ant colony optimization (ACO), neural networks, fuzzy logic, and genetic algorithms for optimizing the network lifetime. Another important performance metric in WSN is energy efficiency. This metric is taken into consideration during the survey of routing protocols in [16] so that the energy is optimized through the use of SI-based data communication protocols in WSN. The authors in [17] focus on the evolution of social activities in different natural creatures such as insects, fish, birds, and honey bees, and a significant range of routing protocols for WSN have been built based on these species' foraging habits. Further, there are some issues in the WSN like clustering, routing, and localization of nodes which are considered as NP-hard problems. The main objective of the research paper in [18] is to present the use of various nature-inspired optimization algorithms to address the WSN challenges. The solution to these network issues will decrease the consumption of battery power and prolong the lifespan of the network. The researchers have presented a critical examination of all optimization methods and use this information to determine possible future directions. It is also learned from the related literature that a significant amount of research work have been accomplished to address the WSN issues with the application of NIO algorithms. Moreover, confidentiality of data that is transferred across the network is also achieved through these nature-inspired optimization methods. Due to the resource constraints in WSN, secure routing in sensor networks is a difficult issue. Furthermore, new nodes continuously joining and exiting the WSN have an effect on multihop routing. In the literature, [19] describes the use of nature-inspired optimization techniques for achieving security in the sensor networks. As a result, biologically based algorithms are examined and improved to address problems that occur in WSN. WSN have performed admirably with ant routing and human self-security schemes. In [20], a trust-based secure algorithm is presented using genetic algorithm. This nature-inspired optimization algorithm has used trust factor of each node to decide about the selection of the node as cluster head. This optimized and secure selection has resulted in energy efficient and secure data routing in the WSN. Another ACO-based NIO protocol for energy efficient and secured data transmission is presented by authors in AOSTEB [21]. The protocol executes in three steps, i.e., cluster creation, creation of multiple paths, and transmission of data from source node to the destination. Similarly, another NIO-based routing protocol based on SI-based PSO algorithm is develop to address the core issue in WSN. The proposed protocol LD^2^FA-PSO [22] uses network model for segment table creation and finite automata for path table creation. The protocol achieves energy efficiency and security during data transmission in the WSN. PSO is used for optimally selecting the route for data communication in WSN.

RETRACTED

From the literature, it is discovered that not much research work is conducted using NIO techniques in the opportunistic routing protocols along with the security aspect of the WSN. Moreover, it is learned from the literature that SI-based methods are the most popular methods which are used by researchers in the recent past. The next section of the paper describes the challenges which are directly associated with the routing in WSN.

## 3. Routing-Related Issues in WSN

Routing is the method of sending data from the source node to the destination node in the sensor network. It is also considered one of the most energy-consuming tasks in the overall operation of the wireless sensor network. If the route chosen during the routing process is not optimal, then this leads to the consumption of sensor node energy. There are many more routing-related issues in the WSN which are discussed in the subsections below.

### 3.1. Energy Usage

In a WSN, energy use [23] is a big problem. The network consumes more resources, in case the path from the node transmitting data to the destination sensor node is not optimal.

### 3.2. Arrangement of Nodes

Another issue that arises from the haphazard distribution of nodes in wireless sensor networks is related to the way the sensor nodes are arranged [24] in the area of observation. For energy-efficient networking and network service, a packet forwarding path must be discovered as nodes are deployed at random.

### 3.3. Accumulation of Data

In certain instances, identical data from different nodes may be collated to remove duplicate and correlated data, which is an essential phase in WSN [25]. Since it reduces the number of transmissions, this method of data aggregation should be promoted for optimal routing in WSN.

### 3.4. Load Balancing

Another problem in a WSN is load balancing [26], which may arise due to an unequal distribution of sensor nodes. To achieve standardized power consumption, sensing and transmitting loads should be spread uniformly among nodes in each cluster.

### 3.5. Latency

The term “latency” relates to the time it takes for data packets to travel from point A to point B. This is a new problem in WSN, as multihop and data aggregation will escalate data transmission latency in certain situations [27].

### 3.6. Network Expandability

Since there are too many sensor nodes in a WSN [28], the possibility of network expansion is a challenge. As a result, the routing algorithm must be able to handle a network that is likely to increase in its size.

### 3.7. Security

Security refers to the measure of ensuring that no malicious node participates in the routing process for transmission of data from the source node to the destination node [23]. It is one of the prominent challenges present in the literature and affects the routing process in case a malicious node has participated in the routing process.

All these above-mentioned issues related to data communication in the sensor network have their impact on the energy consumption of the sensor nodes, and therefore, special caution should be applied in designing routing protocols for WSN. A few of the problems listed above are NP-hard (stochastic), which means they cannot be solved using a deterministic solution. We need some sort of nature-inspired optimization techniques or algorithms to deal with these types of problems. Any optimization techniques come with an objective function to find the right and most desirable solution which would be used to address these stochastic types of problems in the routing. The next section of the paper presents a brief introduction related to two recently developed energy efficient and secure opportunistic routing protocols.

RETRACTED

## 4. Intelligent Opportunistic Routing Algorithm (IOP) and Trust-Based Secure Intelligent Opportunistic Routing Algorithm (TBSIOP)

The challenges associated with the process of routing in WSN are highlighted in the previous section, and the authors of this paper have developed two opportunistic routing algorithms for addressing the issue of energy efficiency and security in WSN.  Algorithm 1, Algorithm 2, [3], and Algorithm 3 [4] are designed for the creation of a forwarder list from the neighbour list, intelligent opportunistic routing, and trust-based secure intelligent opportunistic routing, respectively, in WSN.

The execution of these above-mentioned algorithms resulted in achieving energy efficiency and security of data in the WSN. The next section of the paper provides an overview of swarm intelligence- (SI-) based techniques for optimization of routing in WSN.

## 5. Swarm Intelligence-Based Optimization Techniques for Routing in WSN

There are some problems in the real world that cannot be solved in an absolute manner. These problems are sometimes referred to as NP-hard or stochastic problems. The solution for such types of problems is not available in the traditional deterministic approaches. These problems would be solved with optimization techniques. Routing being one of the NP-hard issues in WSN requires optimization methods for its remedy. The objective function in the optimization techniques is of immense importance. This objective function could offer a single or multiobjective function depending upon the type and requirement of the stochastic problem.  Figure 2 depicts the classification of optimization methods based on the search space. The SI-based optimization techniques are of special interest here as they have been used successfully in the past decade for route optimization in WSN. Swarm behavior [30] refers to the mutual behavior of animals or birds of similar size that congregate or move in a particular direction. Swarms are a kind of animal or bird that adheres to three simple principles: (1) they follow their neighbours' lead, (2) always have a close relationship with their neighbours, and (3) avoid colliding with their neighbours. The algorithms that follow swarm intelligence are explained briefly in the subsections ahead.

RETRACTED

### 5.1. Particle Swarm Optimization

The particle swarm optimization (PSO), which Eberhart and Kennedy [31] developed, is a simulation of birds swarming and fish schooling in quest of food. This technique is a population-based, stochastic, global optimization approach that was developed to be simple in use while still being successful [32]. The PSO has been a highly influential algorithm since its inception in 1995, having been implemented in a broad variety of fields. The PSO simulates the velocity and location of particles as they are on the lookout for food. Each particle's location in PSO represents a solution to the issue. The algorithm allows the use of five significant parameters: the particle's velocity, its current location, the global best particle's position, the actual particle's awareness of its former best location obtained, and the best spot discovered by its neighbour. The location and velocity of the particles are updated with each repetition of the algorithm before it hits the termination state. Similarly, the PSO establishes a knowledge archive that records the optimal objective feature values obtained for each particle participating in the quest operation [32]. The algorithm begins by normalizing the objects known as particles in the search space and then iteratively updates their location and velocity. Another protocol proposed by Prithi and Sumathi [22] is named Learning Dynamic Deterministic Finite Automata (LD^2^FA). This protocol is PSO and finite automata-based pathfinding approach. This protocol also employed a route inspection mechanism for secure routing. MATLAB simulations showed good performance in terms of security and network lifetime.

According to the literature, two critical issues of WSN, i.e., clustering and routing, have been addressed by using PSO. The PSO-based routing protocol is developed by authors in [33] to enhance packet delivery ratio, energy, and network lifetime. Similarly, another routing protocol for WSN which is developed with PSO is presented by researchers in [34]. In this paper, the authors used the PSO technique for creating the cluster of nodes by avoiding nodes left with residual energy. The gravitational search algorithm (GSA) is also used along with PSO in this routing protocol. In [35], the researchers have proposed a routing algorithm that uses neural networks with PSO, to make the WSN scalable. The implementation of this nature-inspired algorithm has ensured security with scalability in the WSN. Therefore, it may be concluded that PSO is an effective algorithm that reduces energy consumption and has a rapid convergence rate in WSN.

RETRACTED

### 5.2. Ant Colony Optimization (ACO)

The ant colony optimization (ACO) algorithm is a well-known algorithm that is frequently used in metaheuristics in the literature. The ACO is a computer simulation of ants moving randomly in the pursuit of food. If the ants locate a food supply, they collect particles of the food, and on returning to their nest, typically through a path with less number of ants, spread some amount of pheromones to alert other ants to their finding. As nearby ants pick up on the smell of the pheromone, they would almost certainly follow the successful ant in obtaining the food supply. This methodology is implemented to determine the close to optimal alternative with a minimum number of hops for data transmission in a wireless sensor network (WSN).

An efficient transmission technique which is based on distance (ODTS) is used with ACO in [36]. This technique is advantageous since it allows for the determination of the shortest path between nodes. It absorbs fewer resources and thereby extends the longevity of the network. In another research work [37], the authors suggested that a novel ACO-based routing algorithm with an operator designated for pheromone updates results in reducing the energy consumption, and this algorithm will evenly distribute lost energy across all sensor nodes in the WSN. This technique decreases the network's total energy demand, thus increasing its lifespan. Another protocol was published by Arora et al. [21] recently called as ACO-optimized self-organized tree-based energy balance (AOSTEB). The AOSTEB [21] showed good performance in terms of network lifetime and other factors like throughput enhancements compared to the existing protocols. The simulations were done on MATLAB, and the results were plotted accordingly. Therefore, it is ascertained from the literature that ACO assists in determining the shortest optimum route for efficient routing and offers rapid convergence. The biggest disadvantage is that it consumes more resources than PSO.

### 5.3. Artificial Bee Colony (ABC)

The artificial bee colony (ABC) algorithm was developed in 2009, and the algorithm was influenced by the action of natural honey bee swarms [38]. The ABC divides bees into three categories: scout bees, onlooker bees, and working bees. Scout bees are all that travel around the quest area looking for answers (food source). Similarly, onlooker bees wait in the hive for the scout bees' update. Employed bees, on the other hand, are bees who engage in food source manipulation after seeing the waggle dance of the scout bees. In this technique, the food source symbolizes a response to the objective function. The amount of fluid in a food supply reflects the solution's consistency [39]. When employed bees carry fluid to the nest, they have three options: go again to accumulate more nectar, follow other dancing bees to a new place, or merely remain in the hive. Due to its ability to quickly escape out of a local minimum, previous research on the ABC has shown that it is extremely helpful in feed-forward artificial neural network testing as well as being quite successful in multidimensional search settings. In general, the ABC algorithm is sluggish in its execution.

RETRACTED

### 5.4. Firefly Algorithm (FA)

The authors in [40] developed this population-based algorithm known as the firefly algorithm which is motivated by the blinking behavior of fireflies. In this algorithm, a group of fireflies collaborates to come up with a solution using radiant glowing, which allows them to develop a solution to problems more effectively. Problem solutions are represented by a firefly, whose sparkles are equal to the consistency of the results they reflect. As a consequence, a sharper light firefly draws the attention of other peers, facilitating more discovery of the solutions. Since the fireflies are unisex, they are drawn to a collaborator with strong intensity of light regardless of gender. The distance between the fireflies will be the reason for their brightness among them. Moreover, in case there is no brighter fly near to any particular firefly, the specific firefly will move randomly.

The FA is easy to set up to work well in multimodal quest settings. It is comparable to the PSO except that the search velocities are not considered in its search for solutions [41]. Conversely, it has a difficult fitness function and relies heavily on the proper parameter setting to produce successful results. Even after producing decent performance, the FA is a sluggish algorithm. This may be attributed to the large number of parameters that the algorithm employs in the quest for solutions.

### 5.5. Bacterial Foraging Optimization (BFO)

The bacterial foraging optimization (BFO) is a branch of swarm optimization motivated by the foraging community of bacteria. Passino [42] was the first to suggest this strategy. This method imitates how bacteria migrate in pursuit of nutrients. The same action is used in the bacterial foraging optimization method, where the bacterium reflects the solution and the sum of nutrients shows the fitness benefit.

RETRACTED

The routing challenge along with the clustering problem in WSN is addressed by the authors in [43]. This algorithm has resulted in enhancement in network life with the decrease in the consumption of energy. This algorithm uses the distance and residual energy of nodes in the fitness function to achieve optimization of the WSN. Another method designed for wearable sensing in WSN is suggested in [44], in which the data is collected with the help of drones and BFO is used for data routing. This method reduces sensor power demand, thus increasing network lifespan. In comparison to PSO and ABC, the BFO is beneficial for optimization and has lower energy usage results.

Therefore, in this section of the paper, nature-inspired optimization algorithms for routing in WSN have been described. All of these swarm-based optimization algorithms are used to address the routing-related challenges in WSN. The next section of the paper deals with the simulation results of the two NIO algorithms and their comparisons with the already developed opportunistic routing protocols, i.e., IOP [3] and TBSIOP [4].

## 6. Performance Analysis and Experimental Results

Performance analysis of IOP [3] and TBSIOP [4] has been compared with existing ACO- and PSO-based routing protocols for WSN, i.e., AOSTEB [21] and LD^2^FA [22], discussed in the literature. Simulation-based experimentation was done on MATLAB, and the results are recorded and plotted accordingly. For experimentation, Intel Pentium core i5 7^th^ generation with a processor speed of 2.50 GHz along with RAM capacity of 8 GB and 64-bit Windows 10 has been used. All the compared protocols are simulated on the same platform to maintain uniform results collection.

### 6.1. Simulation Scenario

For this experiment, 25, 50, and 100 sensor nodes are arbitrarily arranged in an observation region of 500×500 m^2^.  Table 1 presents the simulation settings that opted for this experimentation. The parameters in this table remain the same for all protocols. As additional parameters for a specific protocol for AOSTEB, which is an ACO-based protocol, pheromone and heuristic control factors are considered to be 1 and 2, respectively. For PSO-based protocol, i.e., LD^2^FA, the settings for PSO-specific parameters remain the same. The number of particles has remained as 60, string length was at most 10, a number of loops were 50, and other parameters also remained the same.

For simulation analysis, all the protocols are simulated on the same platform and similar network settings. The other protocol-specific requirements may differ, and the results were recorded accordingly. Base station positioned at the center of the area of deployment and all the nodes will send their packets towards this fixed location only. Protocols under consideration start working instantly after the distribution of nodes. The performance factors considered here are the security of the protocols, energy efficiency, packet delivery ratio, end-to-end delay, and network lifetime. The values for these performance factors are recorded, and the graphs are plotted accordingly.

RETRACTED

### 6.2. Average Risk Level

Figure 3 presents the average risk level which was calculated during the simulation of all protocols. This factor represents the number of malicious nodes encountered during packet transmission. This factor is associated with the disruption in packet transmission. As all the nodes must be used as relay nodes apart from collecting data, malicious nodes will not forward data packets further. This interrupts transmission progress, and path reformation is required. The average risk factor is calculated as a number of such nodes encountered during simulation, where there is a requirement of path reformation. TBSIOP showed good performance due to trust value calculations. Also, LD^2^FA applying secure route inspection for removing various malicious nodes showed performance equivalent to TBSIOP. IOP and AOSTEB do not employ any security measures and ultimately showed poor performance as shown in Figure 3.

### 6.3. Packet Delivery Ratio

The packet delivery ratio for each protocol under consideration is calculated, i.e., the number of packets generated during the simulation and the number of packets successfully received at the base station. The delivery ratio for TBSIOP and LD^2^FA (Figure 4) is almost similar because both the protocols can elude grey-hole and black-hole attacks. These protocols evade both selfish and compromised sensor nodes and reject these nodes from the neighbour list of source nodes. Packet delivery ratio drops drastically for IOP and AOSTEB when the number of malicious nodes increases.

### 6.4. End-to-End Delay

End-to-end delay is another performance parameter that is used to calculate the QoS of the sensor network. This parameter inside the simulation is computed for successfully received packets at the destination. In presence of malicious nodes, end-to-end delay is high for IOP and AOSTEB. This is because these two protocols need to recalculate the path for certain packet transmissions and introduce overhead on the source node. For TBSIOP and LD^2^FA, the end-to-end delay is comparable; however, LD^2^FA involves extra calculations for PSO and needs more time to calculate the secure path as we can see in Figure 5.

### 6.5. Energy Consumption

The importance of calculating energy efficiency is very high in wireless sensor networks as all sensor nodes are energy-constrained. As stated previously, the routing process consumes most of the node's energy, and hence, there is a requirement for energy-efficient routing protocols. TBSIOP considered energy as a factor inside trust factor calculations; the energy consumption for the routing process is distributed among each node of the network except malicious nodes. So, from Figure 6, it can be depicted that TBSIOP showed good performance as compared to other protocols.

RETRACTED

### 6.6. Network Lifetime

Similarly, the network lifetime of TBSIOP as shown in Figure 7 is good, as it is totally dependent on the nodes' available energy. Network lifetime is considered as the time spent on network operations from starting of the network to the first node dead.

## 7. Conclusion and Future Scope

In this paper, a comparative analysis has been presented between IOP, TBSIOP, and nature-inspired algorithms AOSTEB and LD^2^FA-PSO. Analysis of all the protocols was done on a uniform platform, considering the same parameters. Further, during simulation of all protocols, malicious nodes have been introduced for generating grey-hole or black-hole attacks. To launch these attacks, malicious nodes disrupt the packet transmission by dropping packets. Due to this scenario, the performance of network reduces automatically. TBSIOP, a protocol of intelligent lookup for malicious nodes introducing trust factor calculations, has been proved to be the most secure protocol.

Other compared protocols failed to detect attack-generating nodes, and risk factors will be high. The average network lifetime using TBSIOP is highest along with the least energy consumption as compared to other protocols. The average risk level is also lowest in the case of TBSIOP as compared to other compared protocols. Security and energy efficiency are important factors to be optimized by any of the routing protocols to cope with existing challenges with WSN. Nature-inspired algorithms may be used to find the best routes in WSN, but modification is required for improving the network lifetime and security as depicted from the results in this paper. To make routing decisions faster for improving data transmission, the researchers can propose hybrid approaches including trust-based and nature-inspired algorithms. In the future, other swarms of intelligence-based nature-inspired algorithms may be simulated for performance analysis and addressing the possibility of the different types of attacks in the layered network architecture of WSN.

## Figures and Tables

**Figure 1:** Swarm intelligence-based popular techniques for routing in WSN [11].

RETRACTED

**Figure 2:** Nature-inspired optimization algorithms based on search space.

**Figure 3:** Performance based on average risk level.

**Figure 4:** Performance based on packet delivery ratio.

**Figure 5:** Performance based on end-to-end delay.

**Figure 6:** Performance based on total energy consumption.

**Figure 7:** Network lifetime.

**Algorithm 1:** Selection of nodes for the forwarder set (SN=source; DN=destination) //Any time a source node SN wishes to transmit a data packet towards DN, the following steps will be executed.

**Algorithm 2:** Selection algorithm for relay node (SN = source; DN = destination) //when any random sensor node SN wishes to send a data packet toward DN based on the forwarder list that has already been developed.

**Algorithm 3:** Trust-based secure node selection in FDL (SN, DN) **//** Let us assume that SN is ready with the transmission of packets toward DN and it has already made its FDL.

**Table 1:** Parameters for simulation.

Simulation parameter	Value
Area (in square meters)	500 × 500
Number of sensor nodes	25, 50, and 100
Number of compromised nodes (%age of total nodes)	10, 25, and 50
Energy of each node at start (in joules)	2
Electronic energy (Eelec)	50 nJ (50∗0.000000001 joule)
Amplification energy (Eamp) (in joules)	100 pJ (10∗0.000000000001)
Size of packet (in bits)	50
Threshold energy (eth) (in joules)	0.2

## Data Availability

No data has been generated during the study.
